RETRACTED

# Targeting Streptomyces-Derived Streptenol Derivatives against Gynecological Cancer Target PIK3CA: An In Silico Approach

**DOI:** 10.1155/2022/6600403

**Published:** 2022-07-11

**Authors:** H. Jemmy Christy, Swetha Vasudevan, S. Sudha, Mahmoud Kandeel, Kumaran Subramanian, S. R. Pugazhvendan, P. Ronald Ross, Velmurugan

**Affiliations:** ^1^Department of Bioinformatics, Sathyabama Institute of Science and Technology, Chennai, Tamil Nadu, India; ^2^Department of Biotechnology, Sathyabama Institute of Science and Technology, Chennai, Tamil Nadu, India; ^3^Department of Biomedical Sciences, College of Veterinary Medicine, King Faisal University, Al-Ahsa, Saudi Arabia; ^4^Department of Pharmacology, Faculty of Veterinary Medicine, Kafrelshikh University, Kafrelshikh, Egypt; ^5^Centre for Drug Discovery and Development, Sathyabama Institute of Science and Technology, Chennai, Tamil Nadu, India; ^6^Department of Zoology, Arignar Anna Government Arts College, Cheyyar, Tamil Nadu, India; ^7^Department of Zoology, Annamalai University, Annamalai Nagar, Cuddalore, Tamil Nadu, India; ^8^Department of Biology, School of Natural Science, Madda Walabu University, Oromiya Region, Ethiopia

## Abstract

*Streptomyces* is amongst the most amenable genera for biotechnological applications, and it is extensively used as a scaffold for drug development. One of the most effective therapeutic applications in the treatment of cancer is targeted therapy. Small molecule therapy is one of them, and it has gotten a lot of attention recently. Streptomyces derived compounds namely streptenols A, C, and F–I and streptazolin were subjected for ADMET property assessment. Our computational studies based on molecular docking effectively displayed the synergistic effect of streptomyces-derived compounds on the gynecological cancer target PIK3CA. These compounds were observed with the highest docking scores as well as promising intermolecular interaction stability throughout the molecular dynamic simulation. Molecular docking and molecular dynamic modeling techniques were utilized to investigate the binding mode stability of drugs using a pharmacophore scaffold, as well as physicochemical and pharmacokinetic aspects linked to alpelisib. With a root mean square fluctuation of the protein backbone of less than 0.7 nm, they demonstrated a steady binding mode in the target binding pocket. They have also prompted hydrogen bonding throughout the simulations, implying that the chemicals have firmly occupied the active site. A comprehensive study showed that streptenol D, streptenol E, streptenol C, streptenol G, streptenol F, and streptenol B can be considered as lead compounds for PIK3CA-based inhibitor design. To warrant the treatment efficacy against cancer, comprehensive computational research based on proposed chemicals must be assessed through in vitro studies.

RETRACTED

## 1. Introduction

Recent clinical studies have revealed that worldwide cancer incidence and associated mortality rates are raising an alarm in the field of healthcare and medicine [1]. Chemotherapy and radiotherapy are the conventional therapeutic strategies for treating cancer, but in many situations, a focused strategy is lacking, leaving patients exposed to drug resistance. Novel concepts have emerged in recent years to improve existing therapy options for malignancies with poor survival results. [2]. In recent times, the collecting of genomic, transcriptomic, and proteomic data for the structural and functional organization of regulatory processes in a cell has enabled the detection of disease-related traits and the selection of highly promising targets for prospective drug development [3, 4]. Anticancer therapeutics that target apoptosis inhibitor proteins and cancer cell indicators are currently being employed as criterion. Anticancer medicines that are suitable for cancer targets are commonly discovered through in silico investigations [5]. Actinomycetes produce many structurally varied secondary metabolites, many of which have pharmaceutically significant biological activities [6]. Researchers have concentrated their efforts on investigating marine actinomycetes as a source for the search for novel secondary metabolites since these organisms have the most genetic and metabolic diversity [7–9]. Among Actinobacteria phylum, Streptomyces is the most prevalent and productive drug-producing genus [10, 11]. The species can be found in a wide range of environments, including arctic regions, deserts, mountains, insects, plant stems, and marine sediments. This species can be found in a wide range of environments, including arctic regions, deserts, mountains, insects, plant stems, and marine sediments [12]. Streptomyces species have shown a phenomenal potential to deliver secondary metabolites, many of which are used to treat human illnesses. Differential expression studies on a variety of malignancies, as well as allied in silico methodologies, are promising strategies for identifying treatment targets [13]. Polyketides, peptides, and polyketide-peptide hybrids were secondary metabolites of Streptomyces species that have been demonstrated to have therapeutic potential against cancer cells [14]. The cytotoxic activity of streptenol derivatives A, C, F, G, H, and I against cancer cell lines were assessed in the earlier studies. Based on the literature survey, we defined our systematic study to explore the structural scaffolding of the proposed streptenol derivatives. Streptomyces misionensis-BAT-10-03-123, marine-derived bacterium-based stretenol derivatives were tested in cell lines and revealed anticancer activity [15] PI3K elevated activity is often associated with various human cancers and anticancer drug resistance [16, 17]. Phosphatidylinositol-4,5-bisphosphate 3-kinase catalytic subunit alpha (PIK3CA) complexed with alpelisib and the receptor-based pharmacophore model were employed for further virtual screening of the streptenol derivatives as inhibitors for PIK3CA. Streptenol derivative binding mode towards the promising cancer target PIK3CA was studied in the present study. PIK3CA heterodimer catalytic subunits are tightly controlled by the associated regulatory subunits. Although the same p85 regulatory subunits associate with all class IA PI3Ks, the functional outcome depends on pocket specificity of catalytic subunit. In addition, physicochemical and drug-likeness property assessment of compounds and subsequent intermolecular studies to screen their therapeutic efficacy was done using the ligand fit algorithms.

RETRACTED

## 2. Material and Methods

### 2.1. PIK3CA as Promising Player of Cancer Cell Signaling Pathway

The Cancer Genome Atlas (TCGA) project is a collective effort to compile data from a variety of cancer types and make it accessible to researchers across the world. TCGA enabled the comprehensive and coordinated process to accelerate our understanding about the PIK3CA and their molecular level involvement in cancer induction [18]. PIK3CA mutation prevalence was also assessed among the various cancer types and was also recorded. Differential expression analysis was carried out using the GEO2R platform to screen the PIK3CA upregulation among the top listed cancer categories like breast, cervical, and ovarian cancers [19].

### 2.2. Metastasis Profile of PIK3CA among the Cancer

The principal reason for cancer-related death is metastasis, which seems to be the spread of cancer from one organ to another without being directly associated with it. When considering effective treatment techniques for cancer patients, it is vital to evaluate the prevalence of metastasis. At the transcriptional level, a variety of techniques have been used to discover and define genes involved in cancer metastasis. By pooling several data sources, it is crucial to characterize the complex molecular mechanism. Our comprehension of cancer metastasis requires an integrated assessment of multidimensional transcriptome data. CMDB was created to bring these data together and make studying gene expression deregulation in metastasis easier [20].

RETRACTED

### 2.3. PIK3CA Functional Network Assessment Using Gene Multiple Association Network Integration Algorithm

GeneMANIA uses a repository of organism-specific weighted networks to build the consistent set, generate hypotheses regarding gene functions, evaluate gene lists, and prioritize genes for functional studies. PIK3CA Gene MANIA uncovers functionally related genes for the query gene using a multitude of genomics and proteomics data. In this mode, it weights each functional genomic dataset according to its prediction value for the query. Gene MANIA was utilized in this study to depict molecular network analysis to investigate probable PIK3CA linked gene interaction networks and mechanisms [21].

### 2.4. Selection of Streptomyces-Derived Compounds and Structure Retrieval

Based on earlier studies on crude extract isolation from the potent *Streptomyces sps-*based streptenol derivatives that were included for the present study, open-source repository PubMed was used to retrieve the three-dimensional structure and physicochemical attributes of the proposed compounds [22]. The prepare ligand module was used to determine the atom's coordinates and bond order, and then hydrogen was added to the proposed compounds and optimized using CHARMM force fields [23]. Streptenol derivatives were further reduced with the smart minimizer, which used conjugate gradient algorithms and 2000 steps of steepest descent to keep the RMS gradient at 0.001 kcal/mol. For pharmacophore hypothesis creation, fitting of the chemical into the model hypothesis, and affinity evaluation against cancer-related protein targets, minimal conformers were used [24].

### 2.5. Physicochemical and Drug-Likeness of Streptomyces-Derived Compounds

Intermolecular interaction studies of proposed compounds with promising cancer therapeutic target PIK3CA started with three-dimensional structure retrieval of compounds in SDF format from the PubChem database [25]. The SMILES (Simplified Molecular-Input Line-Entry System) notation has been used to analyze the chemical properties and drug-likeness score of three compounds. Lipinski's filter takes into account molecular weight, Clog*P*, polar surface area, number of hydrogen bond donors and acceptors, number of atoms, violations, rotational bonds, and volume [26]. Lipinski rule-based assessment for the derived compounds listed as bioavailability radar in the Figure 1. Drug-likeness is a qualitative notion that describes how a drug reacts to elements like bioavailability and assesses the compound's toxicity. The drug-likeness score of the bioactive compounds was computed using SwissADME, a web resource for efficiently assessing several drug likeness features using a few high-quality prediction models [26].

RETRACTED

### 2.6. Modeling of Pharmacophores Based on Ligands

The Auto Pharmacophore Generation applied on the DS was started to critically probe into the main chemical properties imbibed inside the proposed streptenol derivatives to generate the most feasible pharmacophore models. The information rendered by the above was exploited in the generation of the pharmacophore. The genetic function approximation (GFA) model was used to find the pharmacophore with the best selectivity. Compounds with pharmacophore characteristics were created to test for essential properties that are important for intermolecular interactions with cancer targets [27]. The HypoGen approach, which incorporates the biological activity values of the compounds in the training set and creates the hypothesis on the discovery studio platform, was used to create pharmacophores. To create compound conformers per molecule, the “BEST” algorithm was used.

### 2.7. Receptor-Ligand Pharmacophore Generation (Structure-Based Approach)

To get insight about the receptor-based pharmacophore model generation for PIK3CA-inhibitor complex, experimentally resolved structure (4JPS) was retrieved from the PDB [28]. The structure of PIK3CA was generated by removing the heteroatoms. The presence of PIK3CA residues near the FDA inhibitor alpelisib was investigated and reported. Meanwhile, all other PIK3CA proposed inhibitors and their residue preference were also recorded. Biovia Discovery studio module *Receptor-ligand Pharmacophore Generation* model was created with the help of Pharmacophore Generation. The best pharmacophore model was chosen based on a high selectivity score and appropriate interactions with catalytic active residues of the ATP-binding site PIK3CA. The selectivity score categorizes pharmacophore models based on the sensitivity and specificity of novel ligands against the receptor, with the best models being returned. During the selectivity score computation, the generated pharmacophore models are evaluated to a comprehensive 3D database of drug-like compounds available in DS, and the selectivity is measured using the genetic function approximation (GFA) method. A training set of 1544 pharmacophore models was used to develop the GFA model in DS. Each pharmacophore contains between two and eight pharmacophoric features, which are used to evaluate the CapDiverse database in DS. Descriptors derived from the total number of features in pharmacophore models and interfeatures distance bin values are used to train the GFA model.

### 2.8. Intermolecular Interaction Studies of Bioactive Compounds of Streptomyces

Molecular docking of Streptomyces-derived compounds used to identify their low energy binding mode with the binding cavities of the cancer target receptors. In general, small molecular interaction with the appropriate receptor or target could create an antagonist effect and can be used as a therapeutic agent [29]. In our computational studies, we used the ligand fit algorithm to screen the *Streptomyces-*derived compounds intermolecular interactions [30]. LigandFit docking algorithms used to screen out incompatible ligands and quickly create shape-based alignments of compound poses. They evaluate the volume and shape of the receptor's binding site pattern for screening. The receptor patterning on a grid was used to initiate the binding site analysis for cancer targets. Binding site identification includes two processes like receptor shape-based screening using the Eraser algorithm [31] and volume-based occupancy of ligand posed within the binding cavity [32]. The LigandFit algorithm-based docking approach is divided into two parts: identifying the cavities inside the cancer target receptor as the docking site and docking Streptomyces-derived compounds to the site. Multiple orientations/variation dataset of the ligand key moments with the prime position of the site yield a suitable ligand conformation for the given binding site. Finally, the dock score energy function is used to rank the promising ligand interaction pose with the specified receptor protein.

RETRACTED

### 2.9. Molecular Dynamic (MD) Studies of Streptenol Derivative and PIK3CA Complex

The molecular dynamic simulations have been performed on the CABS Flex 2.0 platform. In recent days, this coarse-grained simulation-based model for assessing protein motion has evolved as a key tool. CABS Flex-based fluctuation plot listed the RMSF values using the Monte Carlo dynamics. Parameters set for 50 trajectory frames within the time span of 10 ns. Distance restraints with global weight of 1.0, and Poisson-Boltzmann/generalized born (PB/GB) molecular mechanics were considered for conformational stability of the PIK3CA-streptenol derivative complex system [33, 34].

## 3. Results

### 3.1. PIK3CA-Key Player of Cancer Cell Signaling Pathway

The high incidence of PI3K pathway mutations in cancer has inspired lots of new therapeutic development efforts addressed in the present study. Despite the fact that numerous robust and specific inhibitors have been developed and tested in preclinical models, clinical licensing has limitations. Mutational landscape of PIK3CA and expression profile data PIK3CA among the various cancers was retrieved from TCGA and depicted in Figures 1 and 2. Differentially expressed PIK3CA profile was retrieved from the GEO dataset and tabulated in Table 1. PIK3CA was listed as top genes among the upregulated expression data of gynecological cancer-related datasets, and the volcano plot depicted their localization in the dataset as in Figure 3.

RETRACTED

### 3.2. Metastasis Profile of PIK3CA among the Cancer

According to the HCMDB, metastasis expression profile data of PIK3CA its revealed that differential expression for PIK3CA is associated with regional lymph node metastasis among the cervical and ovarian cancer patients; in addition, PIK3CA mutation was also associated with metastasis progression among the breast cancer patients and reported data represented as Figure 4.

### 3.3. PIK3CA Gene Network Assessment

The gene-gene interaction network of PIK3CA was assessed using the GENEMANIA platform. Proposed PIK3CA interaction network framed by the GENEMANIA gene function prediction program was based on the Multiple Association Network Integration Algorithm (MANIA), and this systematic algorithm integrates a set of functional features of PIK3CA, like coexpression, pathways, physical interactions, colocalization, genetic interactions, and protein domain similarity. It has been observed that this algorithm is more precise and computationally efficient than other gene function prediction methods as in Table 2. Finally, gene-gene interaction network was visualized in GENEMANIA platform, and the features of the created network were given in Figure 5.

### 3.4. Protein Target Retrieval and Feature Assessment

Experimentally resolved three-dimensional structure of PIK3CA bound with FDA-approved inhibitor alpelisib was downloaded from PDB. In discovery studio platform, the Cavity algorithm was used to rank the listed binding site. Specific amino acids V851, I848, S854, I932, I800, P778, Y836, Q859, M772, D933, and K802 localized in ATP binding pocket 3D structure of PIK3CA were considered as region of interest. The prepare protein module was used to fix common issues such as inserting missing loop regions based on SEQRES data or user-defined loop definitions and calculating the pK and protonation of the supplied PIK3CA structure.

### 3.5. Drug-Likeness and Pharmacophore Feature Assessment

The calculation of pharmacokinetic parameters such as ADMET is an important aspect of the drug discovery process. We used two web resources, namely, SwissADME and Discovery studio ADMET screening, in the currently proposed work and assessed data that was shown in Figure 6. SwissADME is a web platform that estimates physicochemical attributes of streptenol derivatives and includes the pharmacokinetics and drug-likeness assessment of proposed compounds. For lipophilicity prediction, it used numerous extrapolative models and a consensus technique to assess the streptenol derivatives. In this study, ADME analysis was used to see if suggested compounds might make the designated targets, and it was discovered that all the compounds on the list met the drug similarity requirements.

RETRACTED

### 3.6. Receptor–Ligand Interaction Analysis Using Molecular Docking

In gynecological cancers, PIK3CA is the most often mutated oncogene, and somatic mutations in the PIK3CA gene result in enhanced PI3K activity. PIK3CA mutations have been linked to increased cell proliferation and decreased apoptosis in cervical cancer. Five PI3K inhibitors have been approved by the US Food and Drug Administration so far (copanlisib, idelalisib, umbralisib, duvelisib, and alpelisib) (FDA). This has persuaded clinicians and researchers to investigate different PI3K inhibitors in preclinical and clinical settings to find a powerful PI3K inhibitor with significant clinical efficacy, minimal toxicities, and optimal bioavailability. Streptenol derivatives streptenols A, C, and F–I and streptazolin bound resolutely at the PIK3CA cavity by forming conventional hydrogen bonds, C-H bonding, and series of pi-stacked bonds with residues Val 851, Ile 848, Ser 854, Ile 932, Ile 800, Pro 778, Tyr 836, Gln 859, Met 772, Asp 933, and Lys 802 (Tables 3 and 4). Stable conformer of streptazolin mediated the interaction through Pi-stacked bonds with val 850, Met 922, and TRP 780, and key residues like Val 851 and Ser 854 conferred the C-H bonding. Streptenol D similarly conferred a conventional hydrogen bond with Ser 854 and Glu 849 and Trp 780. PIK3CA binding residue Asn 853 and Ser 854 mediated the H-bonding, and Val 851, Tyr 836, Phe 930, Ile 932 conferred Pi stacked interactions with proposed streptenol F, and streptenol B conferred series two Pi stacked interactions with residues Trp 780 and Met 772 and conventional hydrogen bond with Ser 854, Val 8851, and Glu849. PIK3CA residue positions Val 851, Glu 849, and Ser 854 conferred three stable hydrogen bond with streptenol C; similarly, streptenol E also mediated the H-bonding with Val 851 and Ser 854 residues of PIK3CA, and interaction details were depicted in Figure 7. Streptenol I conferred the interactions with Glu 849, Met922, Ile932, and Trp 780 residues of PIK3CA interaction types that are specified in Figure 7. Streptenol G mediated the conventional H-bond with Val 851 and Ser 854 residues and two pi stacked interactions with Ile 848 and Ile 932 of PIK3CA.Streptenol H conferred e hydrogen bond with Val 851 and Arg 852 and Pi-alkyl bond with Ile 932. Reference FDA-approved inhibitor alpelisib also confirms the similar residue preference with PIK3CA, and the interaction details were illustrated in Figure 7. Proposed streptenol derivatives mediated the hydrogen bonding with the druggable cavity residues of PIK3CA. Ser854, Val 851, and Glu 849 were the residues conferred the maximum number h-bond interactions. PIK3CA drug target residue preference towards streptenol derivatives mediates hydrophobic interactions and was shown in Figure 8. PIK3CA drug target ATP binding pocket residues preference towards streptenol derivatives was depicted in Figures 9 and 10. Q849 is not conserved within the PI3K family. Isoforms b, d, and c have an aspartic acid, an asparagine, and a lysine residue, respectively, at this position. The aspartic acid and lysine residues of the b and c isoforms are obviously not able to establish the same hydrogen bond donor–acceptor interactions with the primary amide group of the inhibitor as a glutamine. Q849 mediated hydrogen bonding formed a favorable interaction of the inhibitor with the ATP pocket, but hinge region residue Val 851 is highly conserved among the PIK3 family proteins, and this promising residue mainly mediated the streptenol-based compound interaction; in general, kinase inhibitors target these “hinge-binders” localized in the ATP binding site sits at the interface between the two lobes of the kinase domain.

RETRACTED

### 3.7. Molecular Dynamic Simulation (MDS) Evaluation of the Docked Complex

The receptor employed in this work was PIK3CA, and we examined the binding pocket as well as druggable residues using the cavity method based on literature data. MDS of PIK3CA was carried out using CABSfex2.0 server by 50 ns simulation. Simulation results revealed a fluctuation plot representing the PIK3CA amino acid level fluctuations observed in the phase of simulation. Both svg formatted graphics data and numerical data were recorded for analysis. Residues with higher RMSF values were shown to have greater flexibility, and the details were depicted in Figure 11. Larger RMSF values indicated greater flexibility, whilst smaller RMSF values indicated restricted mobility during simulations. When utilizing effective restraints in the all-atom molecular dynamics' technique, a famous simulation methodology for proteins, the findings demonstrate that there are acceptable secondary structure residues with the -helix and -sheet of the protein that present with little fluctuation. Under all these conditions, proposed streptenol derivatives were displayed to provide their molecular connections with the focus on protein, confirming their potential interaction. Overall, the findings clearly imply that streptenol derivatives could be used as a lead candidate in the development of PIK3CA inhibitors.

RETRACTED

## 4. Discussion

Kinase proteins are implicated in a wide range of biological functions, such as metabolism, cell signaling, protein regulation, cell trafficking, secretion, and many more. Nearly 497 protein kinases were identified in eukaryotes and in those 58 regular kinases well studied for their physiological role. Functional kinases represent 2% of the overall human genome construct, and kinases were first enzymes assessed for their function in oncogenic evolution and considered as potential drug target in cancer therapy [35]. The essential players in gynecological cancer pathways are PIK3CA, BRAF, and epidermal growth factor receptor (EGFR), which are key members in tumor microenvironment. PIK3CA is the second most highly mutated protein reported in cancer studies next to p53. PIK3CA related mutation was observed in 14% of cancers studies and seems to be amplified in 6% of all cancers in their Pan-Cancer Proteogenomic Atlas [36]. Their key physical importance is reflected in pharmacological research, with kinase-related preparations accounting for almost all new drugs discovered today. Kinase domain is localized between the 797 and 1068 residue positions of PIK3CA and was considered as key element and catalyzes substrate phosphorylation; thus, we assessed the proposed compound interaction pattern with this site. Streptomycetes produce a multitude of bioactive secondary metabolites with significant pharmacological potential. More than 60% of today's anticancer/antitumor medications come from these natural sources [37, 38]. Cancer chemoprevention is just as vital as carcinogenesis intervention. Antagonist agents stop the neoplastic process or suppressing agents that inhibit cancer cells from acquiring a malignant phenotype. As a corollary, attempts to find exceptionally accurate and efficient chemotherapy/chemo preventive medicines from other sources such as microbes are progressing [39]. In this research paper, study was designed to find the novel selective allosteric inhibitor for PIK3CA from streptenol derivatives. Anticancer effect of Streptomyces derivatives has a long-term success history, and it started with doxorubicin which has an antibiotic made by the bacteria *Streptomyces peucetius* [40]. Since the 1960s, it has been commonly used as a chemotherapeutic agent. Doxorubicin is a prescription medicine that belongs to the anthracycline group. Methods based on receptors and ligands can be used to create pharmacophore models. The structure of the PIK3CA target complexed with an approved inhibitor was used in our investigations [41]. We analyzed all the experimentally resolved PIK3CA structure complexed with inhibitor before constructing the multiple receptor-ligand based pharmacophore model of PIK3CA inhibitors and further employed the receptor ligand interaction-based pharmacophore technique to reconnoitre the structure activity relationship of proposed cancer drug target PIK3CA and streptenolderivatives. Hydrogen bond acceptor (HBA), hydrogen bond donor (HBD), hydrophobic (HY), negative ionizable (N), positive ionizable (P), and ring aromatic (RA) were among the properties that were considered for the study. Streptenol compounds' projected physicochemical and ADMET properties were within the acceptable optimum standards for medication development [42]. The ADME parameters suggested that proposed compounds with good quality attributes, such as water solubility, human intestine absorption, plasma protein binding ability, and others, were discovered. Furthermore, the molecules streptenol D, streptenol E, streptenol C, streptenol G, streptenol F, and streptenol B were projected to be safe with minimal or no toxicity. Multiple human malignancies have somatic mutations in the phosphatidylinositol-4,5-bisphosphate 3-kinase catalytic subunit alpha (PIK3CA), which encodes the p110 catalytic subunit of PI3K [43, 44]. The ATP pocket is located at 772, 780, 800, 836, 922, 930, 851, 848, 770, 778, 850, 932, and 933, while the non-ATP pocket is located at 954, 955, 956, 957, 1043, 1044, 984, 1047, 1051, 960, 964, 977, 980, and 981 [45]. Alpelisib makes hydrophobic contact with three spine residues (RS4, CS6/8) and the gatekeeper residue (Sh2). The proposed compounds also conferred hydrophobic contact with the first residue of the P-loop M772 and W780 of the *β*2-strand, which make up the specificity pocket [46]. In PIK3CA, hinge residues localized between 849 and 851 were considered as prime region because of their h bonding with ATP especially adenine. Thus, the main objective of present study focused to assess the streptenol derivative interaction with this residue. Proposed streptenol derivatives are found between p110 residues Ile800, Val850, and Val851 on one side and Met922, Phe930, Ile932, and and Asp932 on the other side on of PIK3CA.The docking results revealed that H-bonds and hydrophobic interactions with specific residues such as Val 851, Ile 848, Ser 854, Ile 932, Ile 800, Pro 778, Tyr 836, Gln 859, Met 772, Asp 933, and Lys 802 may play an vital part in the molecular contacts between the streptenol derivatives streptenol D, streptenol E, streptenol C, streptenol G, streptenol F, and streptenol B and the PIK3CA. Ligand binding underpins a wide range of recognition mechanisms that are generally understudied due to a lack of studies using Streptomyces-derived compounds. The application of trustworthy computational approaches to investigate protein–ligand interactions can substantially improve our perception of such systems and advantage to the development of innovative streptenol-based lead molecules for cancer treatment. Proposed compounds as well as reference compound interaction pattern with PIK3CA binding pockets especially hinge region, specificity region, affinity region, and nonconserved region were considered in the present study to support the reference compounds. PIK3CA is a lipid kinase composed of N- and C-lobes, which are connected by a hinge region, and ATP binds to a small pocket between these lobes. The hinge is conserved among PI3Ks, and the ATP-binding pocket residues are key to design the lipid kinase inhibitors. Further in vitro studies will support the present findings.

RETRACTED

## 5. Conclusion

Compared to standard chemotherapy and surgery listed for gynecological cancer, molecular targeted therapies were considered as more specific as well as lesser side effects. Marine-derived bacteria comprise a promising source of new secondary metabolites with diverse chemical structures and interesting biological activities for drug development and particularly, marine actinobacteria represent an attractive resource for anticancer compounds. We performed a comprehensive computational study to identify potential effective inhibitors of PIK3CA from Streptomyces-derived compounds. Spine and shell residues of active PI3K*α* as well as surrounding residues mainly mediate the intermolecular interactions with streptenol derivatives. Our study revealed that streptenol D, streptenol E, streptenol C, streptenol G, streptenol F, and streptenol B can be used as lead compounds in the development of PIK3CA inhibitors. However, further in vivo and in vitro studies are warranted before these drug candidates could enter the market for clinical applications.

## Figures and Tables

**Figure 1:** PIK3CA mutational profile and their prevalence among various cancers.

**Figure 2:** TCGA project-based PIK3CA prevalence among various cancers.

**Figure 3:** Differential expression profile of PIK3CA in various cancers.

**Figure 4:** TCGA derived PIK3CA metastasis-related expression data of various cancers.

**Figure 5:** PIK3CA protein-protein interaction network.

**Figure 6:** Streptenol derivative pharmacophore scaffold and geometrical constraints. The pharmacophore features were colored as follows: green hydrogen bond acceptor (HBA), red hydrogen bond donor (HBD), orange ring aromatic (RA), and cyan hydrophobic (HY).

**Figure 7:** Proposed streptenol derivative intermolecular interaction with the ATP binding pocket residues of PIK3CA.

RETRACTED

**Figure 8:** PIK3CA drug target residue preference towards streptenol derivatives by mediating hydrogen bond interactions.

**Figure 9:** PIK3CA drug target residue preference towards streptenol derivatives by mediating hydrophobic interactions.

**Figure 10:** PIK3CA drug target ATP binding pocket residues preference towards streptenol derivatives.

**Figure 11:** Root mean square fluctuations in protein structures in response to streptenol derivatives:

**Table 1:** Differentially expressed PIK3CA retrieved from GEO dataset.

GEO accession number	Platform	Control	Sample
GSE6791 (cervical cancers and head/neck)	GPL570	56	76
GSE39001(cervical cancer)	GPL201	12	12
GSE22035 (breast cancer)	GPL570	15	15

**Table 2:** Annotated functions of PIK3CA with its interacting proteins/genes based on the protein/gene-protein/gene interaction network.

Function	FDR	Genes in network
Regulation of protein kinase B signaling	7.29*E*-13	10
Protein kinase B signaling	7.29*E*-13	10
Phosphatidylinositol-mediated signaling	1.12*e*-12	9
Inositol lipid-mediated signaling	6.57*e*-12	9
Phosphatidylinositol 3-kinase signaling	3.36*e*-09	7
Regulation of phosphatidylinositol 3-kinase signaling	7.63*e*-08	6
Phosphatidylinositol metabolic process	2.02666*e*-06	6
Receptor tyrosine kinase binding	5.74532*e*-05	3
Phosphatidylinositol 3-kinase complex	5.74532*e*-05	3

**Table 3:** Molecular docking study between streptenol derivatives along with PIK3CA revealed their intermolecular docking scores.

Compound ID	Ligscore Dreiding 1	Ligscore Dreiding 2	PLP1	PLP2	JAIN	PMF	Dock score
11769676-streptazolin	1.34	3.66	50.37	37.05	-0.56	40.84	47.889
132967417-streptenol F	2.34	4.34	68.81	67.67	-1.03	56.76	66.014
10947351-streptenol D	2.89	4.4	70.14	72.76	-0.82	38.44	66.355
15675440-streptenol B	3.21	4.28	71.24	83.57	0.23	44.59	67.926
10921190-streptenol C	1.97	3.53	71.93	77.56	-0.48	34.43	68.057
10609345-streptenol E	2.75	4.43	81.81	78.14	0	58.16	76.359
132967420-streptenol I	1.88	4.8	94.65	93.04	-0.77	68.86	88.275
132967418-streptenol G	1.41	3.49	94.71	95.23	-2.04	69.49	88.432
132967419-streptenol H	2.36	4.49	100.65	95.99	-1.3	76.04	96.081
FDA-approved inhibitor-alpelisib	2.16	4.32	98.59	91.62	-1.1	72.08	95.917

**Table 4:** Molecular docking study between streptenol derivatives along with PIK3CA revealed the kind of interactions and bonding distance and the interacting residues.

Streptenol derivatives	Interacting atoms	Bond distance (A^0^)	Bond type
Streptazolin-11769676	Streptazolin:H19-A:VAL851:O	2.56512	Carbon hydrogen bond
	Streptazolin:H19-A:SER854:OG	2.99151	Carbon hydrogen bond
	A:VAL850-streptazolin	5.09434	Alkyl
	A:MET922-streptazolin	5.21562	Alkyl
	A:TRP780-streptazolin	5.02045	Pi-alkyl
Streptenol D-10947351	A:SER854:OG-streptenol D:O1	3.22236	Conventional hydrogen bond
	Streptenol D:H26-A:GLU849:O	2.0072	Conventional hydrogen bond
	Streptenol D:H14-A:SER854:OG	3.05414	Carbon hydrogen bond
	A:TRP780-streptenol D:C13	5.43126	Pi-alkyl
10921190-streptenol C	A:SER854:OG-streptenol C:O1	2.83465	Conventional hydrogen bond
	Streptenol C:H21-A:VAL851:O	2.55821	Conventional hydrogen bond
	Streptenol C:H23-A:GLU849:O	2.69578	Conventional hydrogen bond
	Streptenol C:H20-A:GLU849:O	1.83534	Carbon hydrogen bond
	A:ARG852-streptenol C:C13	4.48454	Alkyl
132967418-streptenol G	A:VAL851:N-streptenol G:O2	2.88574	Conventional hydrogen bond
	A:SER854:OG-streptenol G:O3	2.75294	Conventional hydrogen bond
	Streptenol G:H42-A:SER854:OG	2.02097	Conventional hydrogen bond
	Streptenol G:H31-A:SER854:OG	2.32419	Carbon hydrogen bond
	Streptenol G:H38-A:SER854:O	2.2941	Carbon hydrogen bond
	Streptenol G:H38-A:SER854:OG	2.89904	Carbon hydrogen bond
	Streptenol G:C22-A:ILE848	4.59251	Alkyl
	Streptenol G:C22-A:ILE932	4.14713	Alkyl
132967420-streptenol I	Streptenol I:H37-A:GLU849:O	2.75816	Carbon hydrogen bond
	Streptenol I:C22-A:MET922	5.35331	Alkyl
	Streptenol I:C22-A:ILE932	5.4146	Alkyl
	A:TRP780-streptenol I:C25	5.1071	Pi-alkyl
132967419-streptenol H	Streptenol H:H40-A:VAL851:O	2.94788	Conventional hydrogen bond
	A:ARG852-132967419:C24	3.50435	Alkyl
	Streptenol H:C25-A:ILE932	4.20838	Alkyl
132967417-streptenol F	A:ASN853:N-streptenol F:O2	3.20635	Conventional hydrogen bond	
	Streptenol F:H26-A:SER854:O	2.42357	Conventional hydrogen bond	
	Streptenol F:H26-A:SER854:OG	2.42369	Conventional hydrogen bond	
	Streptenol F:H15-A:SER854:O	2.32294	Carbon hydrogen bond	
	Streptenol F:H23 A:GLN859:OE1	2.83208	Carbon hydrogen bond	
	Streptenol F:C14-A:VAL851	4.754	Alkyl	
	Streptenol F:C14-A:ILE932	5.02592	Alkyl	
	A:TYR836-streptenol F:C14	3.37793	Pi-alkyl	
	A:PHE930-streptenol F:C14	5.43637	Pi-alkyl	
15675440-streptenol B	A:SER854:OG-streptenol B:O2	3.20635	Conventional hydrogen bond	
	Streptenol B:H26-A:VAL851:O	2.42357	Conventional hydrogen bond	
	Streptenol B:H26-A:SER854:OG	2.42369	Conventional hydrogen bond	
	Streptenol B:H30-A:GLU849:O	2.83208	Conventional hydrogen bond	
	Streptenol B:C13-A:MET772	4.754	Alkyl	
	A:TRP780-15675440:C13	5.02592	Pi-alkyl	
10609345-streptenol E	A:SER854:OG-streptenol E:O1	2.68539	Conventional hydrogen bond	
	Streptenol E:H28-A:VAL851:O	2.72975	Conventional hydrogen bond	
	Streptenol E:H28-A:SER854:OG	3.04873	Conventional hydrogen bond	
	Streptenol E:H29-A:VAL851:O	2.39476	Conventional hydrogen bond	
	Streptenol E:C16-A:ILE848	4.50287	Alkyl	
	Streptenol E:C16-A:ILE932	4.13859	Alkyl	

RETRACTED

## Data Availability

The datasets used and/or investigated during the current study are available from the corresponding author upon reasonable request.
